# SCMAG: A Semisupervised Single-Cell Clustering Method Based on Matrix Aggregation Graph Convolutional Neural Network

**DOI:** 10.1155/2021/6842752

**Published:** 2021-10-04

**Authors:** Haonan Peng, Wei Fan, Chujie Fang, Wenliang Gao, Yuanyuan Li

**Affiliations:** School of Mathematics and Physics, Wuhan Institute of Technology, 430205 Wuhan, China

## Abstract

Clustering analysis is one of the most important technologies for single-cell data mining. It is widely used in the division of different gene sequences, the identification of functional genes, and the detection of new cell types. Although the traditional unsupervised clustering method does not require label data, the distribution of the original data, the setting of hyperparameters, and other factors all affect the effectiveness of the clustering algorithm. While in some cases the type of some cells is known, it is hoped to achieve high accuracy if the prior information about those cells is utilized sufficiently. In this study, we propose SCMAG (a semisupervised single-cell clustering method based on a matrix aggregation graph convolutional neural network) that takes into full consideration the prior information for single-cell data. To evaluate the performance of the proposed semisupervised clustering method, we test on different single-cell datasets and compare with the current semisupervised clustering algorithm in recognizing cell types on various real scRNA-seq data; the results show that it is a more accurate and significant model.

## 1. Introduction

Analysis on the gene expression matrix of the single-cell dataset is the critical step to obtain a single-cell type [1–3]. The categories of cells are already unknown. Detecting the type of each single-cell manually will take a lot of time and money. Then, how to obtain the best results of classification through applying a semisupervised learning algorithm effectively and using the single-cell type as little as possible is a research direction worthy of exploration [4, 5].

The current common semisupervised learning algorithms mainly contain generative semisupervised models [6], self-training [7], collaborative training (Co-training) [8], semisupervised support vector machines (S3VMs) [9], and methods based on graph theory [10, 11]. Generative semisupervised models use the unlabeled data to make an attribution according to the distribution generated by the previously labeled data and modify the previous model parameters to better adjust the decision boundary [12], then iterate this process to optimize the model. Self-training uses existing label data to train a classifier and then uses this classifier to classify unlabeled data to generate pseudolabels or soft labels [13], then develops certain criteria for judging and selects the correct label data from the original pseudolabel data and adds it to the classifier for training, and finally iterates to produce the final classification results. Co-training is a kind of self-training, in which the algorithm assumes that each data can be classified from different perspectives and then uses these classifiers trained from different perspectives to classify unlabeled samples and selects those that are considered credible to be added to the training set. Since these classifiers are trained from different perspectives, they can complement each other and improve the accuracy of the classification. Supervised support vector machines use structural risk minimization for classification [14], and semisupervised support vector machines also use spatial distribution information for unlabeled data [15]. Among them, the selection of decision-making hyperplanes should focus on the place where the distribution of low-density unlabeled data and label data are consistent [16]. However, if this assumption is not true, the spatial distribution information of unlabeled data can mislead decision-making hyperplanes and result in worse performance than when only labeled data is used. In recent years, due to the rise of artificial neural networks [17–19], semisupervised clustering algorithms have made breakthrough progress, among which the label propagation algorithm is one kind based on graph networks [20, 21]. In the label propagation algorithm, the connection between the labeled data and the unlabeled data is found in the training data through the construction of the graph analysis structure. Through the edge-to-edge connectivity, the labeled data flow through the unlabeled data during propagation, then use edge connections between the unlabeled data to obtain new labels and the classification results [22]. Considering that one single cell contains a large number of genes, that is to say, the characteristic dimension of each single cell is extremely high, a single classic classifier cannot learn all the high-dimensional features. Therefore, we consider using a graph convolutional neural network method to deal with high-dimensional complex connections [23–25]. The graph convolutional neural network transfers the similarity between cells to the connection relationship between the edges in the graph and then uses the convolution operation to further extract the classification features of the edges. Due to its powerful feature extraction capabilities, this algorithm shows strong performance in semisupervised clustering. However, the algorithm needs to adjust many parameters in practical applications, especially how to transform the expression matrix of genes on cells to a connection graph that can effectively reflect the similar relationship between cells is a key issue. To solve this problem, we propose SCMAG. The framework of our proposed method is presented in Figure 1. We finally demonstrate that the performance of this algorithm is better than other semisupervised clustering algorithms through tests on different datasets.

## 2. Materials and Methods

### 2.1. Data Description and Data Preprocessing

To verify the effectiveness of the method, we executed four datasets which are summarized in Table 1. These datasets are downloaded from the NCBI Gene Expression Omnibus (GEO) repository (https://www.ncbi.nlm.nih.gov/geo).

The datasets are in the form of a matrix *X*(*g* × *n*), which represents that there are *g* genes in a row and *n* cells in a column. Since the amount of gene expression varies greatly in each single-cell, we use min–max normalization [30] to normalize the data to (0,1):

(1) $$\begin{array}{c} X_{\text{std}}\left(g\times n\right)=\frac{\left(X\left(g\times n\right)-X_{\min\left(\text{axis}=0\right)}\right)}{\left(X_{\max\left(\text{axis}=0\right)}-X_{\min\left(\text{axis}=0\right)}\right)}, \end{array}$$

(2) $$\begin{array}{c} X_{\text{scaled}}\left(g\times n\right)=X_{\text{std}}\left(g\times n\right)\times \left(\max-\min\right)+\min, \end{array}$$

where *X*_min(axis = 0)_ represents the row vector composed of the minimum value in each column, *X*_max(axis = 0)_ is the row vector composed of the maximum value in each column, max represents the maximum value of the interval to be mapped to (the default value is 1), and min represents the minimum value of the interval to be mapped to (the default value is 0). *X*_std_(*g* × *n*) is the standardized result and *X*_scaled_(*g* × *n*) is the normalized result, then we use cosine similarity to measure the relationship between cells [31].

(3) $$\begin{array}{c} H\left(i,j\right)=\frac{X_{\text{scaled}}\left(i,:\right)⊗X_{\text{scaled}}\left(j,:\right)}{\left\|X_{\text{scaled}}\left(i,:\right)\right\|\times \left\|X_{\text{scaled}}\left(j,:\right)\right\|}, \end{array}$$

where *X*_scaled_(*i*, :) represents the *i*-th row of *X*_scaled_(*g* × *n*). ⊗ represents the inner product. ‖*X*_scaled_(*i*, :)‖ is the modulus of *X*_scaled_(*i*, :). *H*(*i*, *j*) represents the value in the *i*-th row and *j*-th column of the similarity matrix *H*(*n* × *n*).

### 2.2. Data Division by Threshold

We divide *H* into multiple different matrices by threshold:

(4) $$\begin{array}{c} K=\left\{K_{t}=0.1\times t,t=1,2,3,4\right\}, \end{array}$$

(5) $$\begin{array}{c} S=\left\{S_{n},n=1,2,3,4\right\}, \end{array}$$

(6) $$\begin{array}{c} S_{n}^{ij}=\left\{\begin{array}{cc} 1, & H\left(i,j\right)\geq K_{t},\\ 0, & H\left(i,j\right)<K_{t}, \end{array}\right. \end{array}$$

where *K*_*t*_ is the threshold, *S*_*n*_ is the incidence matrix after threshold division, and *S*_*n*_^*ij*^ represents the value in the *i*-th row and *j*-th column of the *S*_*n*_, where 1 means that two cells are correlated and 0 means that two cells are not correlated.

### 2.3. Graph Convolutional Neural Network Construction

To construct a graph convolutional neural network, first of all, we should save the incidence matrix *S*_*n*_ as a graph *G*_*n*_(*V*, *E*). We use the DGL package in the Python library to solve it [32]. Where the number of vertices *V*_*n*_(*G*) is equal to the number of cells, the number of edges *E*_*n*_(*G*) is equal to the number of elements in the *S*_*n*_ whose value is 1. Whether the two vertices in the graph are directly connected is determined by the value in the incidence matrix; the value of 1 means direct connection and 0 means no connection. Then, we build a graph convolutional neural network with two hidden layers, and its structure is shown in Figure 2.

According to equation (4), we can get 4 initial graphs of *S*, and we take each *S*_*n*_ as the input. We randomly select 10% of the cell labels as the true labels, and the remaining 90% of the cells have no labels. In the Chu dataset, the input dimension is 1018∗1018, the activation function is ReLU, the hidden layer dimension is 256, the dimension of the final output probability matrix *I*_*n*_ is 1018∗7, and *I*(*i*, *j*) represents the probability that the *i*-th cell belongs to the *j*-th type. Finally, we select *I*_max_(*i*, *j*) = max{*I*(*i*, 1), *I*(*i*, 2), ⋯, *I*(*i*, *j*)} as the output and choose *j* as the type of *i*-th cell.  Table 2 shows the classification accuracy under different epochs and thresholds.

From Table 2, we can see that GCN performs well under 75 epochs. From 75 to 100 epochs, it shows the trend of convergence, and the classification accuracy is close to 90%. Then, we wonder whether there is a way to make full use of different *S*_*n*_ to get better performance.

### 2.4. GCN Based on Matrix Aggregation

To solve this problem, we build a consensus matrix *P* to minimize the distance between different thresholds [33, 34]:

(7) $$\begin{array}{c} P=\min\overset{m}{\underset{t=1}{\sum }}\overset{n}{\underset{j=1}{\sum }}\overset{n}{\underset{i=1}{\sum }}{\left(P_{ij}-S_{t}^{ij}\right)}^{2}, \end{array}$$

where *P*_*ij*_ is the value of the *i*-th row and *j*-th column in the consensus matrix *P*. Due to the high dimension of the matrix, directly finding the minimum distance will cost a lot of time and memory. Since the values of the incidence matrix *S*_*n*_^*ij*^ are all 0 and 1, we can convert the problem of finding the minimum distance matrix *P* between multiple incidence matrices *S*_*n*_^*ij*^ into finding the number of occurrences of 0 and 1 for each *S*_*n*_. We use count_0_ and count_1_ to count the total times of occurrences of 0 and 1.

(8) $$\begin{array}{c} P_{ij}=\left\{\begin{array}{cc} 1, & {\text{count}}_{1}\geq {\text{count}}_{0},\\ 0, & {\text{count}}_{1}<{\text{count}}_{0}. \end{array}\right. \end{array}$$

We take the minimum distance matrix *P* as the input of graph convolutional neural network for training, then we compared it with the current commonly used semisupervised learning methods; under different epochs, the classification accuracy is shown in Figure 3.

On the Chu dataset, we found that the SCMAG showed better performance than other semisupervised methods, and we also compared it with the GCN without matrix aggregation. The result suggests that the accuracy of classification has increased by nearly 5%.

## 3. Experiments and Results

To further demonstrate the performance of the proposed method SCMAG, we apply the Patel, Xin, and Usoskin datasets for testing. We use label propagation, label spreading, self-training, and GCN, four classic semisupervised learning algorithms for training; then, we use SCMAG to compare with the previous four methods. After 25, 50, and 75 iterations, we get the final result, and classification accuracy is shown in Table 3.

Table 3 shows the comparison results for the Patel, Xin, and Usoskin datasets. In the Patel and Xin datasets, while the number of iterations is 25, 50, and 75, the accuracy of the GCN method is higher than that of the label propagation, label spreading, and self-training methods. When the number of iterations is small, the accuracy of the SCMAG method is lower than that of the GCN, but as the number of iterations increases, the accuracy of the SCMAG method gradually approaches and finally exceeds GCN. In the Usoskin dataset, the label spreading method has the highest accuracy after 25 iterations, followed by SCMAG. But when the number of iterations increases, the performance of GCN is better than the previous three methods. It is worth noting that SCMAG has the highest accuracy rate among the five methods. Therefore, SCMAG is the best method for cell identification.

## 4. Conclusion

Single-cell RNA sequencing technology has made a great contribution to the identification of single-cell types, but single-cell datasets often have a large amount of data and high dimensionality. It usually takes a lot of time to identify them. So whether other cell labels can be measured with only part of single-cell data labels is a direction worthy of research. In recent years, some semisupervised learning methods have begun to be used for single-cell data analysis.

In this study, we have proposed SCMAG for the classification of cells. Compared with the conventional graph convolutional neural network, we divide the similarity matrix by different thresholds to get different incidence matrices, and then, we construct a minimum distance matrix, and it can make full use of the high-dimensional information in the cells and better reflect the characteristics of the cells. We also test the cell classification accuracy of several commonly used semisupervised learning methods, label propagation, label spreading, self-training, and normal GCN under the same conditions. We found that SCMAG shows the best average performance in classification accuracy compared to the other four competing approaches.

Although SCMAG makes considerable improvement on identifying cell types, there remains room for improvement. Several problems are still open. For example, when the single-cell dataset contains a large number of cells, it will cost a lot of time to save the incidence matrix as a graph, and the division of threshold is also a question worth studying. In the future work, we will focus on these questions and hope to achieve more promising results.

## Figures and Tables

**Figure 1:** The workflow of the SCMAG. The input is a gene expression matrix; the algorithm includes four steps: (1) the similarity matrix is calculated by the cosine similarity formula; (2) the incidence matrix is judged by the threshold; (3) the consensus matrix is constructed by the matrix aggregation method; (4) the consensus matrix is saved as a graph; (5) lastly, the graph is used as input to the GCN classifier for training.

**Figure 2:** Graph convolutional neural network structure.

**Figure 3:** Accuracy under different methods.

**Table 1:** List of datasets and their attributes.

Datasets	Number of cells	Number of cell types	Number of genes	Number of GSE	References
Chu	1018	7	19097	GSE75748	Chu et al. [26]
Patel	430	6	5948	GSE57872	Patel et al. [27]
Xin	1600	8	39851	GSE81608	Xin et al. [28]
Usoskin	622	4	25334	GSE59739	Usoskin et al. [29]

**Table 2:** Accuracy under different iterations and thresholds.

*K*_*t*_	Iteration			
	25	50	75	100
0.1	50.2	84.7	89.2	88.4
0.2	50.6	82.3	89.7	89.3
0.3	51.4	87.3	89.3	89.4
0.4	62.8	86.6	88.1	87.6

**Table 3:** Performance comparison in different methods.

Dataset	Iteration	Label propagation	Label spreading	Self-training	GCN	SCMAG
Patel	25	50.3	44.6	50.2	62.3	60.4
	50	67.8	59.1	58.5	76.5	75.7
	75	69.6	65.2	61.4	78.3	79.1
Xin	25	70.5	63.4	60.4	74.6	78.9
	50	77.1	74.6	68.2	87.1	90.6
	75	79.8	75.2	72.7	89.6	91.4
Usoskin	25	35.4	39.2	37.5	36.8	38.2
	50	38.1	41.4	43.3	43.7	44.1
	75	41.6	43.2	44.8	44.9	45.2

## Data Availability

The datasets supporting the conclusions of this article are available in the GEO database repository under accession numbers GSE75748, GSE57872, GSE81608, and GSE59739. The Python codes for our SCMAG method are available from the corresponding author on reasonable request.
